# Sustainable Development Research of Green Smart Park in High-End Manufacturing Based on Internet of Things

This article has been retracted.

**DOI:** 10.1155/2022/3961647

**Published:** 2022-09-29

**Authors:** Jinlei Deng

**Affiliations:** College of Economics and Management, Wuhan University, Wuhan, 430072 Hubei, China

## Abstract

During the transition from industrial production to intelligent, there are still a large number of manufacturing industries in the traditional production mode. The problems of slow information transmission, difficult integrated production management, and complicated process parameter control have led to disconnect decision-making from actual production. In addition, the current manufacturing industry is more of a traditional management method, and the upgrade and iteration speed are slow, and it is not combined with the technology of the Internet of Things. Therefore, the purpose of this article is to use the Internet of Things monitoring technology to explore the improvement of high-end manufacturing and analyze the problems and solutions in the process of consistency of ecological environment and economic effects. This article will use the research methods of specific problems and specific analysis to compare the data and draw conclusions. This article will discuss the technical mechanism of the Internet of Things monitoring and introduce the collection and data of production status data of each station equipment in the production workshop during the production process: improving the current production model, learning foreign experience at the same time, quickly carrying out load curve and data center data accumulation on the service capabilities of the park, verifying multiple operating models, and simultaneously exploring new management models. Based on comparative advantage analysis, the study draws similarities and differences in the development of high-end manufacturing industries at home and abroad, learns advanced experience, proposes improved methods and paths, combines new environmental protection paths, and finally proposes energy operation in the park. Build a green and intelligent park to provide a theoretical reference for sustainable development. The research results show that computer monitoring technology and methods have effectively improved the production environment of high-end manufacturing, combined with the development status of the existing ecological and intelligent composite production system; the infrastructure construction of industrial parks in the new era, IT support, services, manpower resources, and industries has developed rapidly.

## 1. Introduction

With the fast grow and in-depth use of new information technology like Internet of things, Internet plus, and AI, people's quality of production and life has been greatly improved, which not only promotes the economic development but also provides technical support for the transformation and upgrading of the economic structure. The current smart parks also focus more on smart logistics and IOT construction but lack quality monitoring and supervision. In order to better elevate the green and high-quality development of manufacturing industry, it is necessary to establish a complete monitoring system. In the organizational structure of the monitoring system in the green smart park, monitoring nodes are arranged according to the actual monitoring needs to ensure that the monitoring of the environment in the area and the collection of data and information can be met. It has made great contribution to the sustainable development of high-end manufacturing green smart park.

In the development process of high-end manufacturing industry, smart park has become a new trend and new requirement for the development of industrial park. With the promotion of comprehensive national strength, we are improving our quality of life step by step. But at the same time, we cannot damage the ecological environment [1, 2]. General Secretary Xi pointed out that green water and green mountains are golden mountains and silver mountains, which proves the attitude towards the relationship between natural environment and economic development at the national level. While pursuing material interests, we should also fully consider the negative impact of manufacturing industry chain on other industries and the environment [3, 4]. In the era of wide application technology, we have realized the connection of things through sensors according to the requirements of human production and operation to realize the monitoring of human production status index [5]. Through production monitoring, the calculation and supervision of each production environment indicator in a specific region will be more convenient to update all production indicators in real time, and further efforts will be made towards the goal of green development. To study high-end manufacturing green smart park, we need to observe and analyze the industrial park, people, and environment as a whole and apply Internet of Things, big data, and cloud technology to improve the level of environmental management [6, 7]. In addition to the data collection function of environmental awareness, that is, the perception of environmental elements becomes more convenient, while accelerating the collection and transmission of information, enriching the methods of data storage and data analysis, it can also cover a wider range, and at the same time, it can build a unified common management data platform [8, 9]. Combined with other big data such as economy, production, life, and business, the comprehensive analysis can bring more perfect decision support to production management [10]. The problem of resources and environment is a common challenge for human beings. As an important carrier of urban economic development, industrial parks must adhere to the concept of green development and enhance their core competitiveness. Accelerating the green development of industry is an important measure to promote the supply side structural reform and promote the stable growth and structural adjustment of industry [11–13].

Since the 1950s, researchers in developed countries and regions have carried out a variety of targeted scientific research experiments on industrial park monitoring and environmental quality improvement [14]. Research at home and abroad shows that a large amount of human and material resources need to be invested in the early stage of monitoring network research and development. European countries are relatively conservative and adopt a monitoring point to collect only one kind of air data information, while the research of the United States in related fields is much more advanced than that of Europe [15, 16]. Many foreign scholars have concentrated on building production quality monitoring networks and national monitoring networks for trial operation of multiple industrial parks, which are used to monitor their production conditions. Then, they conduct professional assessment of air quality in these areas and seek to find their internal change trajectory [17]. Domestic scholars put forward a plan to establish an intelligent environmental monitoring system of the Internet of Things based on the research status of foreign countries. Using 51 single-chip microcomputers as an embedded processor, multiple subnodes collect environmental data through sensors and send it out by wireless module, while the total node receives and displays environmental data wirelessly, and the abnormal environmental data can send alarm SMS through GSM module [18, 19]. By using the data transmission scheme of single-chip microcomputer and GPRS wireless data transmission technology, the hardware connection and software programming of data transparent transmission between serial port and GPRS module are realized. Generally speaking, domestic experts and scholars focus more on the research of the environmental monitoring system of the Internet of Things and cloud computing and propose the establishment of the overall framework of the environmental monitoring system based on the Internet of Things and cloud computing technology [20, 21]. At the same time of gradually strengthening and improving environmental monitoring abroad, China has also completed two stages of important work in environmental protection, from scratch, from low efficiency to high efficiency, from intermittent monitoring to continuous automation, and then to establish its simple automatic monitoring environment network center system [22]. Although our country has made all the achievements in the monitoring of ecological state, there are still many problems in the monitoring of production environment compared with the developed countries, such as insufficient capital investment, backward technology, low accuracy of monitoring module, poor data accuracy, and poor system stability [23]. All of these factors will lead to the stagnation of production status monitoring and also bring some adverse effects on related research work [24, 25]. At present, some areas in our country adopt the traditional manual way to collect data and information. This cumbersome way does not have timeliness and efficiency but also does not meet the requirements of environmental monitoring in actual production, based on the current situation of modern research [26]. In addition, there is relatively little research on environmental monitoring for wireless network communication. At this time, it is of great momentous to develop and design a production environmental monitoring system for the current environmental monitoring work [27]. Chen et al. have constructed a national regional risk indicator system that includes six risk factors and 23 risk indicators. The study found that the three factors with the highest comprehensive weights include the risk of deviation from development, the risk of sustainable development, and the green risk. At the same time, the fuzzy comprehensive evaluation model proposed by the Chen et al. overcomes the shortcomings of the traditional fuzzy comprehensive evaluation model, fully considers the ambiguity and uncertainty of risk evaluation indicators in the context of big data, and also considers the ambiguity of human judgment. However, their research is only a study of one factor of the environment, without taking into account other uncontrollable factors such as policies and natural disasters [28].

Starting from the meaning and traits of the Internet of Things, this paper explores the sustainable development of high-end manufacturing green smart park, expounds the environmental problems brought by the current economic production and construction, mainly existing problems of the industrial park, finds out the reasonable solutions and the balance basis point in line with the monitoring characteristics, and organically combines the two. In the research, the application of the Internet of Things technology to the intelligent monitoring of the park enables the high-end manufacturing industry in the intelligent industrial park to operate more greenly and efficiently. This paper will discuss the mechanism of the monitoring technology and introduce the collection and implementation of the production status data of each station equipment in the production workshop during the production process. Improve the current production mode, learn from foreign experience, quickly carry out the data accumulation of load curve and data center's service ability to the park, verify various operation modes, and simultaneously explore new management mode. Through comparative advantage analysis, this paper studies the similarities and differences in the development of high-end manufacturing industry both at home and abroad, studies advanced experience, puts forward improvement methods and paths, combines the new path of environmental protection, and finally puts forward the experience accumulated based on this mode to explore the optimal mode of energy operation and management in the park, build a green smart park, and provide theoretical reference for sustainable development.

## 2. Method

### 2.1. Core Concepts

#### 2.1.1. Internet of Things

Internet of Things refers to the use of a variety of information collection terminals and information collection technology to obtain all kinds of information needed by the system and through the Internet and other carriers to upload these information data to the processing center for centralized analysis and processing, to get the corresponding results and make reasonable regulatory decisions based on them, and finally to transmit the control instructions to each terminal equipment to achieve intelligent control system. Through radio frequency identification technology and intelligent perception technology, data collection of all elements of the factory workshop, including workers, equipment, materials, and environment, is completed. According to the on-site situation, an appropriate networking mode is formulated, and the information of each station scattered in the workshop is collected and aggregated to the upper computer for processing, so as to realize the monitoring and automatic management of industrial production. In the production supervision of many production workshops, they are often faced with complex working conditions and excessive environmental interference. These environmental factors, as well as the operation status and parameter data of equipment, are the key factors affecting product quality. The use and popularization technology can achieve intelligent scheduling by setting up multiple sensor nodes to collect and supervise the data of idle and working state of the equipment and improve the utilization rate of the equipment; meanwhile, it can also collect the parameter data of the temperature and speed during the operation of the production equipment that will affect the product quality in real time, based on which the production process, and adjust and control the parameters to improve the production efficiency.

#### 2.1.2. Sensor

A sensor refers to a measuring device that can convert the measured nonelectrical quantity into a corresponding quantity of electricity or an electrical parameter output that is easy to handle accurately according to a certain law. According to its basic sensing function, it can be divided into ten categories: heat sensitive element, light sensitive element, gas sensitive element, force sensitive element, magnetic sensitive element, humidity sensitive element, sound sensitive element, radiation sensitive element, color sensitive element, and taste sensitive element. In order to obtain information from the outside world, people must rely on the sense organs. However, people's sense organs alone are not enough to study the natural phenomena, laws, and production activities.

#### 2.1.3. Data Acquisition Technology

Data acquisition refers to the process of automatic acquisition of nonelectricity or electricity signals from intelligent acquisition equipment, such as all kinds of sensors and other devices to be tested and other analog or digital units to be tested. Data collection is the combination and interaction of information technology and physical level. The traditional data collection method is very single. From the initial manual input, equipment supervision, and other manual operation methods to the later development of data collection using collection devices, the low efficiency of the process has been restricting the industrial production. Up to now, the production demand is growing day by day, and the amount of data in production is huge, which brings great difficulties for data collection and data specification and cleaning after it; at the same time, the protocol of industrial data is not standard, including Modbus, OPC, can, control net, PROFIBUS, ZigBee, and other types of industrial protocols, which leads to great difficulties in the interconnection of industrial protocols. The emergence of technology brings great innovation to the methods of data collection, processing, and analysis.

#### 2.1.4. High-End Manufacturing

In different periods and at different levels of social and technological development, the specific manifestations of high-end manufacturing industry are different. The difference in high-end manufacturing is mainly reflected in the way and method of manufacturing, and with the high-end manufacturing, pollution will gradually decrease. Every great change in the field of science and technology has led to a leap in the quality of manufacturing industry: during the first industrial revolution, “high-end manufacturing” means mechanical manufacturing instead of manual manufacturing; during the electrification revolution, large-scale production activities appear and become increasingly mature; “high-end manufacturing” represents the production of electrification and automation; with the popularization and application of computer technology, the production is gradually intelligent and large scale. The advantage of “informatization” is outstanding, which represents the “high-end” manufacturing mode in the new era. From the industrial point of view, the manufacturing industry that is emerging or is likely to develop into an emerging industry, with high technology content, high-added value, and strong market competitiveness of finished products, is defined as high-end manufacturing industry, which is often referred to as “new energy” and “new material” industry. For example, there are “new energy” industries, such as solar photovoltaic industry, marine wind power, and lithium-ion energy storage battery manufacturing, and “new material” industries, such as nanobiomaterials, high-performance carbon fiber composite materials, and additive printing technology.

### 2.2. Research Methods

In the process of monitoring the production status, understanding the production data, comparing with the green standard, gradient lifting tree is one of the excellent methods, which has been widely concerned and applied in industry and other fields. In this paper, the gradient boosting tree algorithm is used to perform deep learning on the monitored video to convert the monitored production status into visual data. In this paper, XGBoost is used as the research method of extreme gradient enhanced tree computing. Based on GBDT, parallel processing is used, and it has high scalability. According to the previous description, boosting, as an efficient algorithm of integrated learning, can adjust the weight of the learning machine according to its performance in the training process, realize the enhancement of weak learning machine, and improve the accuracy of classification. The process is as follows: (1) all training sets are given the same weight; (2) after *n* iterations, each training set is classified by a classification algorithm, and the classification error rate is

(1) $$\begin{array}{c} {\text{err}}_{n}=\frac{\sum \omega_{i}I\left(y_{i}\neq G_{n}x_{i}\right)}{\sum \omega_{i}}, \end{array}$$

where *ω*_*i*_*I* is the weight of the *i*th sample and *G*_*n*_ is the *n*th classifier.

After the iteration, all the classifiers are obtained. From the above steps, it can be seen the classification error samples, whose weight will become higher, in order to optimize the next iteration effect. Finally, the sample is obtained by voting classification results. It is proved by experiments that the loss function of boosting is in exponential form, and the gradient lifting decision tree is to make the loss function drop along the gradient direction in the iteration.

So as to improve the classification accuracy, XGBoost is the optimal implementation of the algorithm. XGBoost model integrates multiple classification regression cart tree models, which are constructed according to different characteristics, and the value of the leaf node of the tree represents the importance of the characteristics. The expression of XGBoost model can be given:

(2) $$\begin{array}{c} \hat{y_{i}}=\overset{K}{\underset{k-1}{\sum }}f_{k}\left(x_{i}\right)f_{k}\in F. \end{array}$$

*K* in the expression refers to the number of cart tree models, *y*_*i*_ refers to the predicted value of a single tree, *x*_*i*_ refers to the *i*th input sample, and *F* refers to the total set of all cart trees with probability in training. XGBoost algorithm does not need to give all the sets of trees but uses gradient lifting method to add a new tree model each time and constantly improves the previous results.

### 2.3. Characteristics of Internet of Things Monitoring

#### 2.3.1. Reflecting Industrial Scale and Production Capacity

Five indicators will be selected, including total industrial output value, number of enterprises, main business income, average number of employees, and production capacity of main products. Among them, the total industrial output value is expressed in the form of currency. The total value of the final products or labor services provided by an enterprise in a certain period of time reflects the total scale and level of production in a certain period of time. The production capacity of main products refers to the core design and manufacturing, application equipment manufacturing, software development and application, system integration, and network operation. The annual production capacity of the five links, such as information service, can be expressed in terms of output value.

#### 2.3.2. Reflecting Industrial Benefits and Development Quality

Five indicators will be selected, including total profit and tax, industrial added value rate, product sales rate, total asset contribution rate, and total labor productivity. Among them, the total profit and tax is an indicator that counts the total profit and tax of the enterprise, which reflects the total profit realized by the enterprise in the quantitative indicator that undertakes the obligation to the region; the industrial added value rate refers to the proportion of industrial added value in the total industrial output value in a certain period of time, reflects the economic indicator that reduces the intermediate consumption, and is also the Internet of Things industry core indicators of development; product sales rate refers to the ratio of sales output value in the reporting period to total industrial output value in the same period, which reflects the extent to which industrial products have been sold and is an important indicator to analyze the balance of production and demand in the Internet of Things industry; total asset contribution rate reflects the relative indicators of the output of total assets of enterprises, reflects the profitability of all assets of enterprises, and evaluates industrial benefit core indicators. The total labor productivity is the comprehensive performance of the production technology level, management level, technical proficiency, and labor enthusiasm of the enterprise, and it is also an important index to assess the industrial efficiency.

#### 2.3.3. Reflecting Innovation Ability and Achievement Transformation

Five indicators will be selected, including R&D expenditure, number of Internet of Things standards, number of patent applications, number of important research results, and sales revenue of new products. Among them, R&D expenditure refers to all kinds of direct and indirect expenses incurred by enterprises in the research and development process of products, technologies, materials, processes, and standards; the number of important research results refers to the number of key technologies that are conquered and recognized by the state in the fields of perception, transmission, processing, application, and other technologies; the new products refer to the research results that are obtained through technological innovation. The product has a breakthrough in one aspect or obvious improvement compared with the original product, thus significantly improving the product performance or expanding the use function, which has a certain part in boosting the economic efficiency of the product and is conducive to the sustainable development of the city's industry.

#### 2.3.4. Reflecting Abnormal Engineering and Development Environment

Five indicators will be selected, including the number of application projects, the number of public service platforms, the number of industrial clusters, the number of key enterprises, and the number of international cooperation. Among them, nonstandard application projects, public service platforms, industrial clusters, and backbone enterprises are all general, standard, independent and controllable application platforms, Internet of Things public service platforms, Internet of Things industrial clusters, and backbone enterprises recognized by the state; international cooperation refers to the establishment of R&D institutions in China and joint R&D and establishment abroad by overseas enterprises and scientific research institutions R&D institutions; this index helps to enhance the international competitiveness of Wuxi Internet of Things industry.

## 3. Experiment

In the experiment of this paper, firstly, the industrial equipment is screened, and the appropriate type of factory equipment is selected, and then, the Internet of Things technology is used to arrange the intelligent monitoring equipment in the factory park. Finally, the intelligent monitoring system is tested.

### 3.1. Data Materials

24 V industrial switching power supply, PLC, temperature and humidity meter, electric energy meter, temperature control meter, pulse generator, Modbus gateway, wire, and other materials are shown in Table 1.

### 3.2. Experimental Test

Assemble the unit data acquisition module, input the PLC's own program, set the slave station address and communication parameters (baud rate 9600, 8-bit data bit, no check bit, 1-bit stop bit) for each instrument connected to 485 bus, check the circuit and power supply safety, and prepare for the subsequent test. As a comprehensive data acquisition and processing module, PLC is an important test object. Firstly, the signal acquisition function and serial communication function of PLC will be tested, and all kinds of instruments will be connected to the corresponding interfaces of PLC (analog input port, digital input port, and serial com port), and then, PLC will be connected through 485 to USB data line direct serial communication with the testing machine computer and data reading and displayed through Modbus poll debugging software. Finally, the test function interface is written through the configuration software, and the data table is read and displayed. The data acquisition and monitoring experiment of the monitoring meter have been completed successfully. The test methods of the temperature inspection instrument, the electric energy meter, and the pulse signal generator are consistent with the above process. After the server and configuration software of the machine room are built, the monitoring screen is projected to the central screen through the remote desktop, so as to realize the production in the workshop site and facilitate the timely supervision and control of the production management personnel.

### 3.3. Purpose of the Experiment

With the widespread use of the Internet, the structural transformation and development of high-end manufacturing industry also need to be improved. Industrial production began to face a series of diversified challenges; the traditional production technology and information management have been unable to meet its development needs. What changed was the birth of diversified integration of the industry, “smart factory,” “smart manufacturing,” and other concepts came out. In this field, centering on intelligent manufacturing, it integrates many technologies such as industrial automation, intelligent logistics, industrial big data platform, and industrial Internet of Things, making manufacturing gradually replaces new blood. Among them, data visualization is very important. Due to the high integration of industrialization and information technology, information technology provides a variety of ways for data collection, such as bar code, two-dimensional code, RFID, industrial sensors, automatic control system, and other technologies that have been fully applied. Through the combination of RF technology and industrial sensors, the data acquisition system covering the whole production system equipment can be realized. At the same time, it is hard to manage a lot of production data only by manpower. Therefore, it is very important to realize data visualization, data centralization, and intelligent control. The intelligent system planning and design of the smart park should take the construction of green buildings and the park as the goal, to achieve functional practicality, timely technology, safety and efficiency, standardized operation, and economic rationality. The intelligent construction planning and design of the park shall be carried out in strict accordance with the building function, building equipment management, building environment management, etc., and the concept of the intelligent park. The planning and design of intelligent monitoring system engineering can know the production status and change the production mode at any time. The intelligent system planning and design of the intelligent park is based on the building and its landscape as the platform, based on the integrated application of various intelligent information, integrating architecture, system, application, management, and optimization, with the integrated intelligent ability of perception, transmission, memory, reasoning, judgment, and decision-making, and providing the park people with a safe, efficient, convenient, and sustainable development function ring environment.

## 4. Discussion

### 4.1. Performance Analysis of Monitoring

#### 4.1.1. Motor Parameter Acquisition Subsystem

Motor parameter acquisition subsystem is the basic measurement unit of the whole motor monitoring system, which is mainly composed of STM32 controller, temperature sensor, voltage, current, vibration sensor, hall speed sensor, LoRa wireless data transmission module, and TFT display interface. Complete the real-time and accurate measurement of the field motor parameters, and transmit the data to the relay data transmission subsystem through the LoRa wireless module, so as to realize the concentration of multiple motor operation parameters. As shown in Figure 1, different aspects of the performance and practicability of the monitoring equipment are affected by the actual application. As shown in Figure 1, in the performance and practicability ratio of monitoring equipment, motor parameter collection, relay data transmission, and data storage monitoring service platform are, respectively, 5.2, 3.2, and 6.7.

#### 4.1.2. Relay Data Transmission Subsystem

The relay data transmission subsystem is the intermediate node of the whole motor condition monitoring system to realize the remote transmission and monitoring of motor data. It is mainly composed of STM32 controller, LoRa wireless data receiving module, and Nb IOT wireless Internet of Things module. Through LoRa wireless module, the wireless local area network function of multiple parameter acquisition subsystems on site is completed, and the data of multiple motor equipment on site is centralized. Then, through the Nb IOT module, the field motor parameters are uploaded to the open platform of the telecom IOT in order to awake the remote networking and data access operation of the field motor data.

#### 4.1.3. Data Storage Monitoring Service Platform

Data storage monitoring service platform is the data storage and remote monitoring interface of the whole motor condition monitoring system. Using the API provided by the open platform of the Internet of Things, the data interaction between the IOT North host computer and the open platform of the Internet of Things is realized, the motor parameters of the front-end parameter collection and transmission unit are acquired, and the acquired parameters are stored in the corresponding data table items of MySQL database. Then, through the remote browser access Tomcat web server, the data in MySQL database is displayed in the remote access end, to achieve the monitoring of the running state of the field motor. As shown in Figure 2, one of the monitoring equipment is the operation of the multifunction peripheral.

### 4.2. Analysis of Monitoring Results

In the parameter setting of quality prediction model based on XGBoost algorithm, some parameters are set as follows, as shown in Figure 3. Each element has different depth and different characteristic performance. The maximum depth of the tree is 5; the number of iterations is 250; the weight sum of the minimum leaf nodes is 5; the random sampling proportion is 0.7; in the selection of the maximum height of the tree, because the height of the tree is too small, the model is too simple, the test performance is not good, and the fitting degree needs to be improved, but when the height of the tree is too large, the model is relatively complex and does not have good applicability, so the maximum height of the tree is set as 6. The adjustment of the number will affect the accuracy, stability, and convergence rate of the model prediction. The depth of tree and the number of trees are two relatively important control parameters. When the number of trees is fixed, the accuracy of algorithm test set will converge to a constant, and with the increase of tree depth, the stability will be greatly improved; similarly, selecting the appropriate number of trees will also enhance the stability of prediction.

The unit data acquisition module equipped with each equipment has basically completed the equipment status data acquisition required by production, completed the communication between the lower sensor and the upper computer through reasonable networking, and successfully implemented the real-time monitoring function through the configuration software. In the real-time data acquisition, there is a slight delay deviation between the actual data of the equipment and the acquisition display data, which has no impact on the product production control within the acceptable range. But it also needs to be improved later. So far, the whole data acquisition and monitoring system have been built, and the equipment number, corresponding IP address, and slave station address are recorded in the upper computer software for later query and management. Configuration software has played its due role. It not only collects and transmits the data of the sensors of the lower equipment but also successfully completes the real-time monitoring of the configuration and provides a variety of monitoring management methods such as trend chart and report form, which provides a good foundation for the subsequent improvement and optimization. In conclusion, XGBoost algorithm has a good performance in quality prediction-oriented classification. In the production process, the prediction model can be used to complete the batch of products according to the existing process parameter settings before they are put into production; the prediction of good product rate has a more comprehensive understanding and control of production and processing, as show in Figure 4.

## 5. Conclusion

As a complex system engineering, the Internet of Things has cross integration with many technologies, such as radio frequency identification, network communication, integrated circuit, computer software and hardware, and system integration. In this technology chain, the backwardness of any link will affect the development of Internet of Things and industry.

Worldwide, Philips, French semiconductor, and Texas Instruments basically monopolize the RFID chip market; Intel, Honeywell, Foxboro, and other enterprises have absolute advantages in the sensor market; IBM, Microsoft, Sybase, Oracle, and other international giants seize the leading position in middleware, Internet of Things system integration, and overall solution market; The core technology of information module and intelligent control equipment is also basically in the hands of European and American multinational companies. As far as China's current situation is concerned, due to the limitation of domestic IC design level, there is a lack of independent intellectual property rights in key core technology areas, which restricts the further development. China has successfully cultivated a number of industry leading enterprises in this field, but in sensor manufacturing, Internet of Things system integration application, public service, and other fields, there is a lack of leading enterprises to control high-end products or core technologies, especially those chain leading enterprises that determine technical standards, master the right to formulate technical standards, and can lead the direction of technological innovation and evolution, which have not yet formed. Effective business model and industrial division system lead to the low output value of the core industry.

Technological innovation and industrial development have the relationship of mutual influence and promotion. At the same time, the development of industry also needs the combination of industrial model matching with relevant technological innovation. With the increasingly extensive application of the technology and the continuous maturity of common markets, the state needs to guide the industry of Internet of Things from support to independence, promote the connotative development of China's Internet of Things industry, achieve technological innovation and surmount in key technologies, and promote the development of new urbanization with greater advantages.

## Figures and Tables

**Figure 1:** Proportion of performance practicability of monitoring equipment.

**Figure 2:** Monitoring equipment of compound machine.

**Figure 3:** Ranking of feature importance.

**Figure 4:** Relationship between XGBoost prediction accuracy and the number of trees.

**Table 1:** Collection and monitoring of plant equipment.

Equipment type	Device name	Equipment number	IP address	From station number
Monitoring computer	Monitoring computer		172.17.7.3	Master station
	Composite machine	JD013	172.17.1.2	1
	Composite machine	JD014	172.17.1.3	2
	Wet compound machine	JD037	172.17.1.4	3
	Wet compound machine	JD039	172.17.1.6	4
	Multifunctional compound machine	JD069	172.17.1.10	5

Slitting machine	Double axis high speed slitter	JD057	172.17.1.17	6
	Double axis high speed slitter	JD058	172.17.1.18	7

Embossing machine	Aluminum foil embossing machine	JD048	172.17.1.14	8
	Aluminum foil embossing machine	D063	172.17.1.27	9
	Aluminum foil embossing machine	D074	172.17.1.22	10

## Data Availability

The data that support the findings of this study are available from the corresponding author upon reasonable request.
